This article has been retracted.

# Green production and green technology for sustainability: The mediating role of waste reduction and energy use

**DOI:** 10.1016/j.heliyon.2023.e22496

**Published:** 2023-11-19

**Authors:** Changlin Li, Sayed Fayaz Ahmad, Ahmad Y.A. Bani Ahmad Ayassrah, Muhammad Irshad, Ahmad A. Telba, Emad Mahrous Awwad, Muhammad Imran Majid

**Affiliations:** a School of Social Sciences, Yunnan University of Nationalities, Kunming, 650031, China; b Department of Engineering Management, Institute of Business Management, Karachi, Pakistan; c Department of Financial and Accounting Science, Middle East University, Amman 11121, Jordan; d Department of Management Sciences, University of Gwadar, Pakistan; e Department of Electrical Engineering, College of Engineering, Kind Saud Univerity, Riyadh, Saudi Arabia; f Department of Electrical Engineering, College of Engineering Sciences, Institute of Business Management, Karachi, Pakistan

**Keywords:** Green production, Green technology, Waste reduction, Energy use, Sustainability, Manufacturing industry

## Abstract

The study investigates the relationship between green production, green technology, waste reduction, energy use, and sustainability. A Partial Least Squares Structural Equation Modeling (PLS-SEM) approach was used for analysis. The data was collected from a sample of companies in the textile industry. The results suggest that green production and technology positively and significantly affect waste reduction and energy use, which mediates the positive relationship between these two factors and sustainability. This study concludes that green production and technology are critical drivers of sustainability and emphasizes the need to prioritize waste reduction and energy use in sustainable manufacturing practices. The study has practical and managerial implications in all production or manufacturing industries and provides a guideline for managers and policymakers to ensure sustainability.

## 1 Introduction

As the global population continues to grow, the demand for natural resources and energy is also increasing at an unprecedented rate [1,2]. To fulfill their needs, manufacturing industries are also continuing to grow with different types of technology and practices. However, this rapid growth through resource utilization and energy consumption also significantly strains the environment, leading to increased pollution levels, greenhouse gas emissions, and waste production [3,4]. Energy and resources are two of the most critical elements for economic development. Without enough resources and energy, economic development is not possible, and therefore, it is necessary to utilize resources and energy wisely and efficiently [5]. Pakistan has been dealing with energy crises for decades, which has resulted in the country's premature deindustrialization. South Asia also has the highest electricity tariffs [6]. Due to this, economic development is possible and threatens sustainability through the use of resources (fossil fuels). The buying and utilization of those fuels again create economic and environmental problems. The power generation installed capacity in Pakistan is 399772 MW as per the National Electric Power Regulatory Authority's report 2021, where thermal (fossil fuels) account for 63 % of energy, hydro accounting for 25 %, renewable accounting for 5.4 %), and nuclear accounting for 6.5 % [7]. Statistics show that household consumption of electricity is about 47 %, commercial consumption is 7 %, industrial consumption is 28 %, agricultural consumption is 9 %, and other consumption is 8 % [8] that leads to carbon footprint and environmental pollution. Another issue is solid waste production as Pakistan reports that 87 thousand tons of solid waste is produced each week, mostly in large cities. Karachi, Pakistan's biggest metropolis, produces around 16,500 tons of municipal waste every day. 18 % ash, bricks, and dirt, 6 % glass, 2 % textile, 7 % cardboard, 30 % food waste, 1 % leather, 6 % paper, 9 % plastic, 1 % rubber, 4 % metal, 2 % wood, and 14 % yard trash [9]. To minimize the impact of these challenges, many industries and individuals are adopting green production (GP) and green technology (GT) to reduce waste and energy consumption (EC), and promote sustainability.

GP and GT use environmentally friendly technologies and production processes to reduce waste and EC and ensure sustainability [10,11]. Such activities and technologies minimize environmental impact, conserve natural resources, reduce carbon footprints during production [12], and minimize EC, which leads to the conservation of natural resources and sustainability [3,13]. Although many researchers have focused on the mentioned variables individually [14,15], the gap exists because they are not studied in a single research. To fill the gap, this study intends to develop a conceptual model for the study, draw relationships among variables, and draw conclusions based on the data collected from employees working in manufacturing industries. This study aims to find the role of GP and GT in waste reduction (WR) and EC. In addition, it is also investigating the role of GP and GT in promoting sustainability by removing waste and energy use. The research seeks to answer the following questions.

1. Is there any relationship between GP and GT towards sustainability?
2. Is there any relationship between WR and EC towards sustainability?
3. Do WR and EC mediate the relationship between GP and GT toward sustainability?

The study has significant importance in examining the present-day economic and sustainability concerns. It aims to clarify the complex relationship between the adoption of green technologies and green industrial practices in light of a growing focus on sustainability around the world. Additionally, it looks at the important mediating components of energy efficiency and waste reduction, which are essential for attaining sustainable environmental goals. The research can provide a guide for companies, governments, and industries to adopt greener policies, reduce waste, improve energy efficiency, and eventually advance sustainability, all of which will contribute to a sustainable future.

GP, GT, WR, and EE are essential elements for sustainability as the function together to advance environmental and economic stability, reduce adverse ecological impacts, and facilitate appropriate utilization of resources. GT provides ecologically favorable alternates, and GP reduces resource use, waste, and carbon emissions. Resource conservation and a decrease in pollution rely on WR while EE reduces emissions and consumption of energy. A green and environmentally friendly future depends on those practices as they promote resource conservation and respect for the environment and society.

## 2 Theoretical framework and hypothesis development

### 2.1 Theoretical framework

The development of the theoretical framework is based on three main theories; Diffusion of Innovation Theory (DIT) [16], Resource-Based View (RBV) [17], and Circular Economy Theory (CET) [18]. The DIT stresses social impact and perceived advantage for the adoption of GP practices and technologies in the industry. The RBV emphasizes the importance of eco-friendly production methods and technology for textile companies, and sustainable competitive advantage. The CET supports resource efficiency and a closed-loop system to reduce waste and increase value creation, which is in line with WR efforts in the textile sector.

*Resource-Based View (RBV):* Green technology and GP processes are important assets that support the company's sustainability and competitive position in the textile sector [17]. They can attract eco-conscious consumers through the implementation of GP practices and green technologies. Energy-efficient technology and WR techniques, help businesses cut expenses, lessen their negative environmental effects, and improve their reputation as responsible companies. It can be concluded that companies adopting green technology and production methods will achieve sustainability and competitive advantage.

*Diffusion of Innovation Theory:* This theory explains how GP techniques and green technology are necessary to be adopted in the textile sector. It explains variables that affect the adoption of green practices, including perceived advantages, compatibility with current systems, complexity, observability, and social impact [16]. Textile companies will implement WR and energy-efficient practices when they see cost savings, enhanced environmental performance, and compliance with sustainability criteria. Moreover, social influence speeds up the diffusion process as businesses observe advantageous results obtained by early adopters of environmentally friendly manufacturing techniques and technology.

*Circular Economy Theory:* CET is aligned with aspects like WR and energy use reduction during the GP process [18]. Textile companies may reduce waste production and increase resource longevity by putting circular economy concepts into practise, like recycling, etc [18]. Resources are conserved and waste is reduced by adopting WR techniques including recycling dye sludge, fabric remnants, and packaging materials which contribute to the aim of the circular economy.

### 2.2 Green production

Green production or green manufacturing is the upgradation of production or manufacturing processes in an environmentally friendly manner [19]. GP minimizes the negative environmental impact and conserves natural resources through environmentally friendly practices [20]. It involves the entire production process, from raw materials to the final product [21]. This includes using renewable resources, energy-efficient processes, and recycling waste materials [22,23]. GP reduces the environmental impact of manufacturing while still meeting the demands of consumers and maintaining profitability for businesses [24]. Examples of GP practices include using recycled materials in manufacturing [25], designing products with a longer lifespan [26], reducing EC during production [27], and using renewable energy sources [28]. The literature shows that GP is one of the main sources of obtaining sustainability through reducing waste during manufacturing, reducing EC and carbon emissions, enhancing recycling or reusing waste or products, and using renewable resources for production.

#### 2.2.1 Green production and waste reduction

GP reduces waste production during manufacturing [29] and minimizes the negative environmental impact [30]. GP minimizes waste production through efficient and renewable resources and consumes as little material as possible [31]. It employs non-toxic materials and implements safer and more secure manufacturing procedures and green practices that reduce hazardous waste [32]. GP uses recycled raw materials [33] and designs products that are recyclable or capable of reuse [34]. It has optimized manufacturing processes [35] that use materials and energy efficiently, decreasing waste and negative environmental impact [36]. Therefore, industries must employ GP technologies and practices to ensure sustainability and a safer earth.

#### 2.2.2 Green production and reduction of energy use

GP reduces energy use and decreases the environmental impact of manufacturing by reducing EC [37] and boosting the use of renewable energy sources [31,33]. Some of the most common ways GP reduces energy use are by using energy-efficient technologies during manufacturing [35], using renewable energy sources, and optimizing production processes relying on energy [38]. These practices lower industrial energy usage and carbon impact on the environment while saving money and enhancing profits [39]. Therefore, it is concluded that GP and the EC are closely related, and the energy issue can be resolved through GP, ensuring sustainability.

#### 2.2.3 Green production and sustainability

Green production strives to reduce the environmental effects of manufacturing while also promoting sustainability [40]. GP uses green technology [41] and methods to reduce energy usage [42], minimize waste [43], and the carbon footprint of production activities in the industry [44]. Production firms can ensure sustainability through the implementation of green practices that reduce carbon footprint and minimize waste disposal and EC expenses [[44], [45], [46], [47], [48]]. Therefore, production industries must use green technology and ensure their production is green and enhance sustainability [10].

### 2.3 Green technology

The concept of Green Technology (GT) is becoming popular with each passing day. Production and manufacturing industries are adopting this technology [[49], [50], [51]]. It is

the tool to produce products, processes, and services that are environmentally friendly and promote sustainability [52]. It assists in the reduction of environmental issues such as climate change, pollution [53], and resource depletion [54] while also supporting economic growth and social well-being [55]. GT encompasses a wide range of fields, including renewable energy, energy conservation [56], clean transportation [47], water and waste management [57], sustainable agriculture, and green building design. Some examples of green technology include solar panels, wind turbines, electric vehicles, energy-efficient lighting, green roofs, and water conservation systems [58].

The benefits of GT include reduced greenhouse gas emissions [59], reduced dependence on fossil fuels, improved air and water quality, and conservation of natural resources [54]. It also produces economic opportunities [55], such as job creation in the renewable energy industry, and reduces business expenditures through energy-efficient products and processes [60]. In short, it is crucial in promoting sustainability and addressing environmental challenges driving economic growth and improving quality of life.

#### 2.3.1 Green technology and waste reduction

Green technology reduces waste production during production and manufacturing, promoting sustainability [49,57]. GT includes adopting environmentally friendly technologies and methods to develop long-lasting products [58], whereas WR tries to reduce the quantity of trash produced during the production process [61]. With the help of GT, industries minimize waste generation, promote green energy [56], lower their carbon footprint [59], and enhance their reputation as environmentally responsible businesses. Green technology also generates economic opportunities, such as developing jobs in the recycling and repurposing industries, and enhances market competitiveness [62].

#### 2.3.2 Green technology and energy reduction

Green technology and energy use reduction are also closely linked to promoting sustainability [63] and reducing the environmental impact of production by reducing EC [64] and encouraging the use of renewable energy sources [56]. Companies that apply these practices can reduce their energy use, lessen their carbon impact [59], and save money on energy prices. GP has the potential to reduce energy usage significantly [64] while also fostering sustainability in production [65,66]. Therefore, it is necessary to use green technology for production activities and ensure the least possible energy use.

#### 2.3.3 Green technology and sustainability

Green technology promotes ecologically friendly practices and seeks to reduce the environmental impact of manufacturing [49]. It is the application of environmentally friendly technologies and processes to generate sustainable products. Industries that adopt green technologies lessen their environmental impact, reduce their carbon footprint [59], enhance green energy [56], and reduce the depletion of natural resources [54] while promoting long-term sustainability. GT practices improve the environment and give economic benefits [60], such as lower waste disposal and EC expenses [55]. Therefore, it is the need of the day to adopt and implement GT in industries to reduce waste and carbon footprint [53] etc. and obtain sustainability [11]. Therefore, the production and manufacturing industries must implement and adopt GT and promote sustainability.

### 2.4 Waste reduction and sustainability

Production or manufacturing processes always produce some waste [67]. To ensure sustainability, waste production must be reduced to the possible level [[68], [69], [70]]. WR is the employment of techniques and technology types to minimize waste output in a manufacturing or production process [71]. It focuses on promoting environmentally-friendly practices and minimizing the environmental impact of manufacturing [72,73]. Hence plays an essential role in promoting sustainability [74]. For example, recycling and reusing [71], a reduction in the utilization of resources [75], and an increase in the efficiency of the production process are some of the important factors that ensure WR [76]. In contrast, WR reduces the consumption of resources such as raw materials and energy, contributing to the conservation of natural resources [77]. WR also reduces the environmental impact of manufacturing by reducing carbon emissions and other liquid and solid leftovers that lead to pollution [78,79]. Efficiency can be achieved through WR, which also reduces production costs and enhances profitability [80,81]. Through reusing and recycling materials, WR assists in conserving resources [82,83]. All these factors promote sustainability without jeopardizing future generations' needs.

### 2.5 Energy use and sustainability

Energy shortage is one of the leading global issues, and most countries face it [84,85]. It runs the industries, and without the EU, development is impossible. Its use cannot be stopped but can be managed to ensure sustainability [86]. Some ways in which the EU can assist in achieving sustainability are by using energy-efficient technologies for production and manufacturing and the use of renewable sources of energy [13,87]. EU is the energy consumed during manufacturing or production [88]. An efficient EU consists of environmentally-friendly practices that reduce the environmental impact of manufacturing [89]. Manufacturing firms must reduce EC to the possible level to promote and maintain sustainability. It also involves optimizing the manufacturing process and the least possible resource consumption [90,91]. With the help of these practices, industries can reduce environmental impact, carbon footprint, and manufacturing costs and promote sustainability.

### 2.6 Sustainability

Sustainability means fulfilling the current generation's needs without compromising the future generation's, ensuring a balance between economic growth, environmental care, and social well-being [92]. It seeks the utilization of natural resources in a way to causes less damage to the environment [93]. Protecting or conserving natural resources, reducing waste production, promoting renewable energy, optimizing the production process of goods and services, producing products in an environmentally friendly manner, and preserving biodiversity are some of the important sustainability practices [94]. It is not against economic development but emphasizes using resources, EC, and WR to ensure as little environmental harm as possible [95,96]. Economic development is associated with the production or manufacturing industries [97]. These industries are significant EC, waste production, and resource consumption sources. Therefore, it is necessary to use energy and other resources very carefully to reduce waste and preserve the environment. GP and GT are the two main factors used in industries that can reduce EC, resource utilization, and waste production, leading to sustainability [10,11]. GP and GT play a critical role in promoting sustainability through the conservation of natural resources, as they ensure their efficient use and reduce waste, which provides their availability for future generations [3,13]. GP and GT promote producing and using renewable energy like wind, solar, etc., which minimizes carbon emissions [12]. GP and GT enable the production and consumption of products and services in an environmentally friendly manner to preserve biodiversity [98,99]. In short, it is the responsibility of individuals, governments, and firms to design, develop, and implement production processes and technology that promote the utilization of natural resources in an environmentally friendly manner. Sustainability can be ensured through the adoption of GP and GT.

### 2.7 Theoretical mechanism, hypotheses, and conceptual model

The theoretical mechanism of the research is based on DIT, RBV, and EIT. It stresses how the use of GP and GT, supported by WR and EE can improve sustainability in today's technological and competitive era. It investigates the complex relationships between GP and GT towards sustainability, having an emphasis on the mediating roles played by EC and WR. According to the RBV, GP and GT serve as important internal capacities for companies. By adopting such practices and technologies, a firm can utilize its resources in a manner to obtain sustainability. Similarly, DIT provides insights for firms to integrate GP and GT in their processes. GT, such as energy-efficient technology is integrated with green manufacturing techniques, environmentally friendly materials, and WR tactics. In other words, DIT provides an understanding of the need to adopt and promote sustainable solutions in the form of GT and GP. In this framework, energy efficiency and WR play an essential part as mediators. Adoption of GP and GT consequently promotes WR and effective usage of resources, following the CIT. Because waste is reduced while resources are preserved under the circular economy framework. The theoretical mechanism leads to the minimization of negative environmental effects and supports sustainability through WR, consuming less energy and having a smaller environmental effect. Firms that effectively pursue this approach acquire a competitive edge by employing the DIT and the RBV principles. Eventually, by reducing waste and maximizing energy efficiency, the mechanism reinforces the concepts of the CET. Companies that take this approach may preserve resources while enhancing economic growth simultaneously. Based on these important theories, the integration of GP and GT, mediated by WR and EE, underlines a commitment to sustainability. Based on this theoretical mechanism the following hypotheses were formulated and the theoretical framework was developed as shown in Fig. 1 which illustrates the relationships between the study's variables.

1. GP has a positive relationship with WR.
2. GP has a positive relationship with sustainability.
3. GP has a positive relationship with energy use reduction.
4. GT has a positive relationship with WR
5. GT has a positive relationship with sustainability.
6. GT has a positive relationship with energy use reduction.
7. WR has a positive relationship with sustainability.
8. Energy use reduction has a positive relationship with sustainability.
9. WR mediates the relationship between GP and sustainability.
10. WR mediates the relationship between GT and sustainability.
11. Energy use reduction mediates the relationship between GP and sustainability.
12. Energy use reduction mediates the relationship between GT and sustainability.

**Fig. 1:** Theoretical framework.

## 3 Methodology

The study is based on a quantitative methodology. Using stratified random sampling, primary data was collected from engineers and managers working in Pakistan's textile industries. Close end questionnaire using a 1–5 Likert scale was used. The data collected includes 600 responses, from the textile industry of Pakistan through a close-ended questionnaire and tested for reliability, convergent validity, discriminant validity, Fornell Larcker Criteria, HTMT analysis, hypotheses testing, model fitness, model robustness, MGA analysis, and importance-performance matrix. The questionnaire was adopted from prior researchers and tested for reliability and validity. PLS-SEM was used for the analysis of the data. Table 1 shows the details of the instruments used in the study.

**Table 1:** Measurement instruments.

Green Production [100]	The company's manufacturing process effectively reduces the emission of hazardous substances or waste.
	The manufacturing process of the company recycles waste and emissions that allow them to be treated and re-used;
	The manufacturing process of the company reduces the consumption of water, electricity, coal, or oil;
	The manufacturing process of the company reduces the use of raw materials.
Green Technology [100]	Green Technology effectively reduces the emission of hazardous substances or waste.
	The company's green technology recycles waste and emissions, allowing them to be treated and reused.
	The company's green technology reduces the consumption of water, electricity, coal, or oil.
	The manufacturing technology should be selected to reduce the use of raw materials.
	Green technology is energy efficient.
	Green Technology effectively reduces the emission of hazardous substances or waste.
	The green technology of the company recycles waste and emissions that allow them to be treated and re-used;
	The green technology in the company reduces the consumption of water, electricity, coal, or oil.
Waste Reduction [101]	The containers of the solutions or materials used in your manufacturing should bear warning labels.
	The waste of your industry needs to be treated before it leaves your facility.
	You believe that changes should be made to your technology to reduce waste.
	You believe that the waste should be recycled for production and use.
	You believe eco-friendly technology can reduce waste.
	You believe eco-friendly production can reduce waste.
Energy Use Reduction [102]	Energy consumption is necessary to be very efficient in manufacturing industries.
	Ecofriendly technology should be used for the reduction of energy use.
	Ecofriendly production should be used for the reduction of energy use.
	Renewable energy sources are good options for manufacturing and sustainability.
	You believe energy saving is important.
	Energy consumption is necessary to be very efficient in manufacturing industries.
	Ecofriendly technology should be used for the reduction of energy use.
Sustainability [103]	We actively monitor water usage in our facilities.
	We actively monitor energy usage in our facilities.
	We implement a systematic approach to setting environmental targets.
	We implement a systematic approach to achieving environmental targets.
	We actively monitor water usage in our facilities.
	We actively monitor energy usage in our facilities.

### 3.1 Data collection

Data were collected from Pakistan's textile industry. After obtaining consent, respondents were asked about their awareness of GT and GP and requested to participate in the study. Only those who understood GT and GP were included. Educational level was also considered during data collection to ensure good results. Stratified random sampling was employed in the data collection process.

### 3.2 Participants

The survey was conducted in textile which is Pakistan's biggest industry. Among the 600 respondents, 400 were male, and 200 were female. Most respondents were graduates, i.e., 500 and 100 were postgraduate. Table 2 shows the descriptive statistics of the study sample.

**Table 2:** Descriptive statistics.

Gender	Number	Percentage
Male	400	66.60 %
Female	200	33.30 %
Total	600	100.00 %
**Education**	**Number**	**Percentage**
Graduate	500	80 %
Postgraduate	100	20 %
Total	600	100.00 %

### 3.3 Reliability and convergent validity

The outer loadings can measure the strength of the connections among items and their related constructs. They demonstrate how accurately each construct "measures" its concept. If the value is higher than 0.5, it is considered a strong indicator. The range of outer loading (0.698–0.872) shows that all items are significantly associated with their constructs. The values show that the study's items effectively measure the relevant constructs. Reliability or internal consistency is measured through composite radiality statistics. If the value is higher than 0.7, it is considered a strong indicator. The results show that the value ranges from 0.82 to 0.91, an acceptable reliability range. It is concluded that the constructs used in the study are reliable and internally consistent. Variance is measured by the average variance extracted. If the value is high, the relationship of items with the construct becomes stronger. It is considered a good indicator if the value equals or exceeds 0.6. The statistics (0.765–0.911) show that the items of each construct are related to their intended one more strongly than to the other constructs. The details are given in Table 3.

**Table 3:** Reliability and convergent validity.

Constructs	Items	Outer loadings	CA	CR	AVE
Energy Use Reduction	ER1	0.848	0.879	0.911	0.672
	ER2	0.821			
	ER3	0.872			
	ER4	0.831			
	ER5	0.72			
Green Production	GP1	0.775	0.765	0.848	0.583
	GP2	0.844			
	GP3	0.73			
	GP4	0.698			
Green Technology	GT1	0.835	0.865	0.9	0.644
	GT2	0.829			
	GT3	0.799			
	GT4	0.833			
	GT5	0.711			
Sustainability	SS1	0.741	0.733	0.825	0.542
	SS2	0.807			
	SS3	0.732			
	SS4	0.658			
Waste Reduction	WR1	0.788	0.873	0.908	0.666
	WR2	0.85			
	WR3	0.898			
	WR4	0.708			
	WR6	0.825			

### 3.4 Discriminant validity

The Fornell-Larcker criterion is a method for assessing the discriminant validity of construct measures in SEM and is indicated by the diagonal values. Table 4 shows higher diagonal values than the correlation, indicating a good discriminant validity for each construct.

**Table 4:** Fornell Larcker criteria.

	Energy Use Reduction	Green Production	Green Technology	Sustainability	Waste Reduction
Energy Use Reduction	0.820				
Green Production	0.019	0.764			
Green Technology	0.464	0.203	0.803		
Sustainability	0.170	0.421	0.144	0.736	
Waste Reduction	0.759	0.004	0.451	0.219	0.816

Discriminant validity can also be assessed through heterotrait-monotrait ratios of correlations. The threshold value for HTMT is 0.9, and the value below this value shows good discriminant validity among the constructs, as given in Table 5.

**Table 5:** HTMT.

	Energy Use Reduction	Green Production	Green Technology	Sustainability
Green Production	0.149			
Green Technology	0.485	0.289		
Sustainability	0.257	0.468	0.267	
Waste Reduction	0.868	0.113	0.493	0.276

### 3.5 Hypothesis testing

Hypothesis testing is a significant statistical tool to assess the viability of research hypotheses. The main objective of hypothesis testing is to determine if a sample's results are statistically significant. It is important because it enables researchers to conclude the population from a small sample of data, reducing the need to study the full population. Additionally, it enables investigators to decide impartially and objectively based on empirical facts and to ensure that the findings are reliable and robust. The summary of hypotheses testing is given in Table 6. The tested conceptual model is illustrated in Fig. 2.

**Table 6:** Hypothesis testing.

Hypothesis	Beta	T-Values	P-Values	Results
*H1: Green Production - > Waste Reduction*	0.091	2.720	0.007	***Supported***
*H2: Green Production - > Sustainability*	0.457	12.750	0.000	***Supported***
*H3: Green Production - > Energy Use Reduction*	0.078	2.010	0.045	***Supported***
*H4: Green Technology - > Waste Reduction*	0.469	14.723	0.000	***Supported***
*H5: Green Technology - > Sustainability*	0.921	3.450	0.000	***Supported***
*H6: Green Technology - > Energy Use Reduction*	0.480	12.897	0.000	***Supported***
*H7: Waste Reduction - > Sustainability*	0.162	2.527	0.000	***Supported***
*H8: Energy Use Reduction - > Sustainability*	0.326	12.339	0.000	***Supported***
*H8: Green Production - > Waste Reduction- > Sustainability*	0.015	2.048	0.041	***Supported***
*H10: Green Technology - > Waste Reduction- > Sustainability*	0.076	2.698	0.007	***Supported***
*H11: Green Production - > Waste Reduction- > Sustainability*	0.015	3.234	0.000	***Supported***
*H12: Green Technology - > Waste Reduction- > Sustainability*	0.076	2.439	0.015	***Supported***

**Fig. 2:** Tested model.

***GP has a positive relationship with energy use reduction:*** The results indicate that the relationship between GP and energy use reduction is negative with a t-value of 2.01, p-value of 0.045, and beta coefficient of −0.078. In other words, an increase in the GP will decrease energy use.

***GP has a positive relationship with sustainability*:** The results show that the relationship between GP and sustainability is positive and significant with a t-value of 12.75, p-value of 0.000, and beta coefficient of 0.457. In other words, an increase in the GP is linked with increased obtaining sustainability.

***GP has a positive relationship with WR:*** The results indicate that the relationship between GP and WR is negative with a t-value of 2.720, p-value of 0.007, and a beta coefficient of −0.091. In other words, an increase in the GP is associated with decreased WR.

***GT has a positive relationship with energy use reduction:*** The results show that the relationship between GT and energy use reduction is positive and significant with a t-value of 12.897, p-value of 0.000, and beta coefficient of 0.480. In other words, an increase in the GT is linked with an increase in energy use reduction.

***GT has a positive relationship with sustainability:*** The results indicate that the relationship between GT and sustainability is positive with a t-value of 3.45, p-value of 0.000, and beta coefficient of 0.921. In other words, the increase in the GT is linked with increased obtaining sustainability.

***GT has a positive relationship with WR*:** The results show that the relationship between GT and WR is positive and significant, with a t-value of 14.723, a p-value of 0.000, and a beta coefficient of 0.469. In other words, the increase in the use of GT is linked with an increase in WR.

***WR has a positive relationship with sustainability:*** The results show that the relationship between WR and sustainability is positive and significant, with a t-value of 2.527, a p-value of 0.000, and a beta coefficient of 0.162. In other words, an increase in WR is linked to obtaining sustainability.

***Energy use reduction has a positive relationship with sustainability*:** The results show that the relationship between energy use reduction and sustainability is positive and significant with a t-value of 12.3, p-value of 0.000, and a beta coefficient of 0.326. In other words, an increase in the reduction of energy usage is linked with increased obtaining sustainability.

***WR mediates the relationship between GP and sustainability:*** The results show that WR mediates the relationship between GP use and sustainability is positive and significant with a t-value of 2.048, p-value of 0.041, and a beta coefficient of 0.015. In other words, an increase in GP will impact WR, resulting in increased obtaining sustainability.

***WR mediates the relationship between GT and sustainability:*** The results show that the WR mediates the relationship between GT and sustainability is positive and significant with a t-value of 2.698, p-value of 0.007, and a beta coefficient of 0.076. In other words, increasing GT will impact WR, resulting in increased obtaining sustainability.

***Energy use reduction mediates the relationship between GP and sustainability:*** The results show that the energy use reduction mediates the relationship between GP and sustainability is positive and significant with a t-value of 2.324, p-value of 0.000, and a beta coefficient of 0.015. In other words, an increase in GP will impact energy use reduction, resulting in increased obtaining sustainability.

***Energy use reduction mediates the relationship between GT and sustainability:*** The results show that the energy use reduction mediates the relationship between GT and sustainability is positive and significant with a t-value of 2.439, p-value of 0.015, and a beta coefficient of 0.076. In other words, an increase in GT will impact energy use reduction, resulting in increased obtaining sustainability.

### 3.6 Model fitness

Model fit is an advanced test used in the SmartPLS to estimate the accuracy of the model of the study. After the items and construct reliability and validity, it is necessary to confirm how their combined structure is valid and fit to estimate the phenomenon of interest. There are several measures used in the SmartPLS to estimate the model fitness like the SRMR, NFI, and Chi-Square etc. according to social science researchers and statisticians, SRMR is the most robust technique to estimate the model fitness in the case of a complex model in SmartPLS. The threshold value for the SRMR is 0.08 or less. Statistics in Table 7 shows the SRMR value of 0.079, less than the threshold value of 0.08, indicates that the model has achieved its fitness.

**Table 7:** Of model fitness.

SRMR	0.079
d_ULS	2.717
d_G	0.745
Chi-Square	2562.469
NFI	0.699

### 3.7 Model robustness/unobserved heterogeneity

There are different measures used for the robustness of the model of a study, but the FIMIX test of the unobserved heterogeneity is the most robust technique when we analyze a complex model based on primary data in SmartPLS. Unmeasured (unobserved) differences between study subjects or samples connected to the (observed) variables of interest are referred to as unobserved heterogeneity. The presence of hidden variables raises the possibility that statistical conclusions from the available data are misleading. The technique used for the unobserved heterogeneity deduction in the SmartPLS is FIMIX. There are three main measures in FIMIX to estimate the unobserved heterogeneity. These measures are AIC3, CAIC, and EN. Suppose the above three measures show a value declining from segment one onward. In that case, this shows that there is not any evidence of unobserved heterogeneity, and the data is homogenous. Table 8 of FIMIX fit indices for the one to four segments shows that all the values in the relative segment are declining, indicating no unobserved heterogeneity in the data. From this, it was confirmed that the robustness of the model was achieved.

**Table 8:** of Fit indices for the one-to four-segment solutions.

Criteria	Segment 1	Segment 2	Segment 3	Segment 4
AIC3 (Modified AIC with Factor 3)	4777.986	4550.657	4044.941	3339.124
CAIC (Consistent AIC)	4826.588	4652.28	4199.584	3546.787
EN (Entropy Statistic (Normed))		0.53	0.703	0.828
Sum	9604.574	9203.467	8245.228	6886.739

### 3.8 MGA analysis

Multi-Group Analysis (MGA) is an advanced technique in SmartPLS that measures the impact of the variation on the relationship of the studies based on the two categories of a group. Simply put, it will explain any change due to the change in the different categories of the study population.

#### 3.8.1 MGA based on gender

The below table of MGA analysis based on gender shows the variation in the relationship of the data based on the male and female. Six hundred respondents’ data was used, among which 400 were males, and 200 were females. The measure used to identify the variation in the relationship is the p-value of a relationship. The threshold value for the p-value is 0.05 or less. Table 9 that all the relationships have insignificant p values indicating that there are not any variations in the relationships of the model based on gender.

**Table 9:** Of MGA analysis based on gender.

Relationships	β-diff (Male-Female)	p-Value
Energy Use Reduction - > Sustainability	0.088	0.575
Green Production - > Energy Use Reduction	−0.003	0.961
Green Production - > Sustainability	−0.069	0.335
Green Production - > Waste Reduction	−0.025	0.740
Green Technology - > Energy Use Reduction	−0.046	0.569
Green Technology - > Sustainability	0.034	0.735
Green Technology - > Waste Reduction	−0.048	0.476
Waste Reduction - > Sustainability	0.016	0.886

#### 3.8.2 MGA based on educational level

Table 10 shows the variation in the relationship of the data based on the graduate and postgraduate. Six hundred respondents’ data was used, among which 500 were graduates, and 100 were postgraduates. The measure used to identify the variation in the relationship is the p-value. The threshold value for the p-value is 0.05 or less. The below table shows that all the relationships have insignificant p values indicating that there are not any variations in the relationships of the model based on academic qualification.

**Table 10:** Of MGA analysis based on educational level.

Relationships	β-diff (Postgraduate - Graduate)	p-Value
Energy Use Reduction - > Sustainability	0.024	0.897
Green Production - > Energy Use Reduction	−0.055	0.501
Green Production - > Sustainability	0.076	0.3
Green Production - > Waste Reduction	0.041	0.619
Green Technology - > Energy Use Reduction	0.05	0.52
Green Technology - > Sustainability	0.083	0.387
Green Technology - > Waste Reduction	0.032	0.623
Waste Reduction - > Sustainability	0.013	0.913

### 3.9 Importance-performance matrix analysis

The importance-performance matrix analysis indicates that energy use reduction has the highest performance, with a value of 72; GT has a performance value of 71; WR has a value of 66; and GP has a value of 56. Higher values indicate higher performance, as given in Table 11. The findings indicate that the firms should concentrate on raising GP's performance, as respondents rated it as the most significant factor, despite having the lowest performance rating. Additionally, firms should keep putting a high priority on GT and energy use reduction, which received high ratings. Finally, as WR is evaluated poorly compared to the other aspects, the firms must reevaluate its perceived importance. Fig. 3 shows the importance-performance map of the variables.

**Table 11:** IPMA analysis.

	Importance	Performances
Energy Use Reduction	0.028	72.002
Green Production	0.455	56.198
Green Technology	0.287	71.805
Waste Reduction	0.108	66.121

**Fig. 3:** Importance-Performance Map.

### 3.10 Q-square

Q-square measures the predictive relevance and shows the dependent variable (endogenous construct) variance accounted for by the independent variables (exogenous constructs). Table 12 of Q-square analysis shows values of 0.142, 0.111, and 0.138 for energy use reduction, sustainability, and WR, respectively. The values indicate that the independent variables moderate the proportion of variance in the dependent variables. Similarly, the Q-square value for GP and GT is 1, which shows that they fully account for the dependent variable variance. The model offers moderate to high predictive relevance for the variables studied.

**Table 12:** Q square.

	SSO	SSE	Q^2^ (=1-SSE/SSO)
Energy Use Reduction	3065	2628.566	0.142
Green Production	2452	2452	
Green Technology	3065	3065	
Sustainability	2452	2180.707	0.111
Waste Reduction	3065	2642.946	0.138

## 4 Discussion

The study's findings show that GT, GP, WR, energy use, and sustainability are positively and significantly related. By implementing these practices, manufacturing industries can considerably lessen their environmental effect, save natural resources, cut operational costs, and promote sustainability. Other studies also support these findings [64]. GP lowers waste by improving production methods and encouraging resource efficiency. E.g., lowering the quantity of raw materials utilized in production or improving energy efficiency can significantly reduce the waste generated. Many other researchers have also had similar results [29,104,105]. According to the results, GP also significantly decreases energy usage and reduces waste. By implementing energy-efficient technology and procedures, industries may minimize energy use and lower carbon footprint. Industries become more profitable while also reducing the negative effects of manufacturing on the environment. Previous studies have also shown such results [[106], [107], [108], [109]]. The finding also clarifies that GP is also directly linked with sustainability. Many previous researchers have also had the same findings [[110], [111], [112], [113]].

Similarly, GT supports sustainability by encouraging appropriate quantity of resource use and minimizing adverse environmental effects. By encouraging sustainability and future growth, these practices assist businesses in creating more robust and long-lasting industry models while promoting sustainability. Many other studies also have similar findings [[114], [115], [116], [117]]. GT and the reduction of waste also go hand in hand. By adopting green technologies, industries can lessen the amount of waste they generate and the adverse impacts of their operations on the planet. For instance, industries can reduce energy usage and carbon dioxide emissions by employing energy-efficient machinery and procedures. Recycling can also help support the circular economy while decreasing waste generation. Previous studies have also observed the same results [115,118,119]. WR, energy use, and sustainability can all benefit greatly from applying GT and GP [113]. People and businesses should adopt these practices to promote environmentally friendly actions like reducing waste production during manufacturing, efficient energy usage, and promoting sustainability [116]. The results also show that waste and EC reduction mediate the associations between GP and GT toward sustainability. Industries may optimize resource utilization, lower operating expenses, and boost competitiveness by lowering waste and energy use production. These factors encourage industries to adopt environmentally friendly technologies and productivity techniques, resulting in more sustainable industry models [[120], [121], [122], [123]]. To achieve sustainability, WR and EC reduction can be very important mediators in the associations between green productivity practices and green technologies. Such measures are critical to promoting sustainable business practices, minimizing the adverse impacts of company operations on the natural environment, and fostering long-term sustainability. By implementing these procedures, firms can increase their competitiveness, optimize resource utilization, lower operational expenses, and create a more sustainable future [[123], [124], [125]].

### 4.1 Research implication

The research findings suggest that sustainable practices must be embraced in the manufacturing sector. Theoretical, practical, and policy implications of the study are given below.

Theoretical Implications.

1. Theories Integration: The study integrates three sustainability theories and shows the impact of their integration and application for understanding the dynamics of GP, technology adoption, WR, and energy use in the textile industry. It focuses on the necessity of considering many theoretical viewpoints to thoroughly analyze and handle sustainability concerns.
2. Mediating Role of WR and Energy Use: The mediation of energy use and WR is another main aspect of the framework that adds a greater understanding of a process by which GP practices and technology impact sustainability performance. This emphasizes how important are waste management and energy efficiency for sustainability.

Practical Implications.

1. Adoption of GP Practices and Green Technologies: To improve their sustainability performance, the study pushes textile firms to embrace GP techniques and technology. Industries can lessen their impact on the environment, save resources, and increase cost-effectiveness by incorporating WR initiatives and energy-efficient technology into their operations. This will result in more market demand for textile goods that are ecologically friendly, higher competitiveness, and improved reputation.
2. Collaboration: Cooperation among textile producers, governmental agencies, academic institutions, and consumers, is crucial for advancing sustainability in the textile industry. It will promote innovation, stimulate the use of green manufacturing techniques and technologies, and build an environment that is conducive to the achievement of SDGs.

Policy Implications.

1. Supportive Policy Frameworks: The study shows the importance of encouraging legislation that encourages GP and green technological advancements in the textile sector. These regulations can foster an atmosphere that encourages sustainable growth.
2. Capacity Building and Education: Policies should also focus on capacity building and educational initiatives to improve the knowledge and expertise of experts in the textile sector regarding GP and technology.

### 4.2 Limitations and future work

The study has some limitations also, which could be considered in future studies.

1. The results may vary across different industries, regions, and organizational contexts. The same model can be tested for other industries and regions.
2. Other factors may be added to the model to present a more comprehensive model for achieving industry sustainability.

### 4.3 Alignment with the achievement of sustainable development goals

The study has significant importance for the attainment of SDGs for tackling global issues and advancing sustainable development across social, economic, and environmental dimensions agreed by the UN in 2015. The following is the summary.

1. SDG 3 (Good Health and Well-being): By lowering pollution, boosting the quality of water and air, and reducing exposure to hazardous materials, GP and GT may enhance public health. This is in line with SDG 3 of Good Health and Well-being.
2. SDG 7 (Affordable and Clean Energy): In line with SDG 7, GT and GP encourage the use of renewable energy sources including solar and wind power. Industries can help increase access to affordable and sustainable energy by cutting energy use and implementing greener energy substitutes. This is aligned with SDG 7 of Affordable and Clean Energy.
3. SDG 11 (Sustainable Cities and Communities): GP and GT are strongly linked with urban areas. Cities may become eco-friendlier, and habitable by adopting WR, and energy-efficient technology which is aligned with SGD 11 of Sustainable Cities and Communities.
4. SDG 12 (Responsible Consumption and Production): GP and GT assist in achieving the concept of a circular economy, where resources are used wisely, waste is reduced, and recyclable goods. This is in line with SDG 12 of responsible consumption and production.
5. SDG 13 (Climate Action): To combat climate change, GT and GP can be used to cut emissions of carbon dioxide and waste. Industries can greatly help to achieve the objectives mentioned in SDG 13 by reducing waste creation and adopting energy-efficient practises.
6. SDG 17 (Partnerships for the Goals): Collaboration is needed among governments, corporations, civil society organizations, and other stakeholders to achieve the SDGs, and GP and GT provide chances for collaborations that encourage sustainability, and knowledge-sharing, and motivate joint action.

## 5 Conclusion

The study examines the associations between GP, GT, WR, EC, and sustainability. The results show positive and significant effects of GP, and GT on Sustainability. Similarly, GP and GT are also positively related to energy efficiency and WR. In addition, the mediating role of energy efficiency and WR is also positive and significant. The findings show that industries must invest in GP, GT, and WR processes, and energy use reduction to promote and ensure sustainability [116]. The results have many theoretical, practical, and managerial implications. The study assists researchers in further enhancing research on other industrial factors to ensure sustainability. Further, it promotes investments in green practices and innovation, which enhance sustainability. Last but not least, it provides guidelines for managers to promote sustainable practices and operations in industries through the adoption of GP and GT.

## Funding

The study was funded by 10.13039/501100002383King Saud University through Researchers Supporting Program number (RSPD2023R1108), 10.13039/501100002383King Saud University, Riyadh, Saudi Arabia.

## Data availability statement

Data will be made available on request.

## CRediT authorship contribution statement

**Chang Lin:** Writing – review & editing, Supervision, Methodology, Conceptualization. **Sayed Fayaz Ahmad:** Writing – original draft, Project administration, Conceptualization. **Ahmad Y.A. Bani Ahmad Ayassrah:** Writing – review & editing, Methodology, Investigation. **Muhammad Irshad:** Methodology, Formal analysis. **Ahmad A. Telba:** Software, Methodology, Data curation. **Emad Mahrous Awwad:** Resources, Investigation, Funding acquisition. **Muhammad Imran Majid:** Writing – review & editing, Validation, Resources.

## Declaration of competing interest

The authors declare that they have no known competing financial interests or personal relationships that could have appeared to influence the work reported in this paper.
